The article "Ultradeep sequencing detects GNAQ and GNA11 mutations in cell-free DNA from plasma of patients with uveal melanoma" was published in 2013. Journal: Cancer Med.

# Ultradeep sequencing detects GNAQ and GNA11 mutations in cell-free DNA from plasma of patients with uveal melanoma

**DOI:** 10.1002/cam4.61

**Published:** 2013-02-14

**Authors:** Claudia HD Metz, Max Scheulen, Norbert Bornfeld, Dietmar Lohmann, Michael Zeschnigk

**Affiliations:** 1 Department of Ophthalmology, Faculty of Medicine, University Duisburg-EssenEssen, Germany; 2 Department of Internal Medicine, West German Cancer Center, Faculty of Medicine, University of Duisburg-EssenEssen, Germany; 3 Institute of Human Genetics, Faculty of Medicine, University Duisburg-EssenEssen, Germany; 4 Eye Oncogenetic Research Group, Institute of Human Genetics, Faculty of Medicine, University Duisburg-EssenEssen, Germany

**Keywords:** Biomarker, cell-free DNA, *GNAQ*, ultradeep sequencing, uveal melanoma

## Abstract

Elevated levels of cell-free DNA (cfDNA) are frequently observed in tumor patients. Activating mutations in exon 4 (R183) and exon 5 (Q209) of *GNAQ* and *GNA11* are almost exclusively found in uveal melanoma, thus providing a highly specific marker for the presence of circulating tumor DNA (ctDNA). To establish a reliable, noninvasive assay that might allow early detection and monitoring of metastatic disease, we determined the proportion of *GNAQ* or *GNA11* mutant reads in cfDNA of uveal melanoma patients by ultradeep sequencing. Cell-free DNA from 28 uveal melanoma patients with metastases or extraocular growth was isolated and quantified by real-time polymerase chain reaction (PCR) (7–1550 ng DNA/mL plasma). *GNAQ* and *GNA11* regions of interest were amplified in 22 of 28 patients and ultradeep sequencing of amplicons was performed to detect even low proportions of mutant reads. We detected Q209 mutations (2–38% mutant reads) in either *GNAQ* or *GNA11* in the plasma of 9 of 22 metastasized patients. No correlation between the proportion of mutant reads and the concentration of cfDNA could be detected. Among the nine ctDNA-positive patients, four had metastases in bone, whereas no metastases were detected in the 13 ctDNA-negative patients at this location (*P* = 0.025). Furthermore, ctDNA-positive patients tended to be younger at initial diagnosis and show larger metastases. The results show that ultradeep amplicon sequencing can be used to detect tumor DNA in plasma of metastasized uveal melanoma patients. It remains to be shown if this approach can be used for early detection of disseminated tumor disease.

## Introduction

Uveal melanoma is the most common primary intraocular tumor in adults 1. Molecular analyses have revealed that there are two distinct classes of this tumor. This knowledge is of clinical relevance because metastasizing disease, which affects 50% of patients, almost exclusively originates from tumors that belong to only one of these classes 2,3. The latency period of uveal melanoma metastases is highly variable, and the preferred site of metastasis is the liver 4. In some patients, metastases have become evident more than 15 years after successful treatment of the primary tumor 5. No effective treatment options for metastatic disease are known, and therefore, prognosis of patients with metastases has remained poor 6. Liver function tests including ultrasound imaging of the liver and detection of lactate dehydrogenase, alkaline phosphatase, and gamma glutamyl transpeptidase have been used to detect metastatic disease 6,7. However, there is no study showing that these markers permit reliable preclinical detection of metastatic disease in uveal melanoma patients.

Serum and plasma of cancer patients as well as healthy individuals are known to contain cell-free DNA (cfDNA) 8. Although already identified in the 1940s by Mandel et al., analysis of cfDNA has lagged in the following decades due to the absence of sensitive and suitable methods of cfDNA detection 9,10. Until now, controversial opinions exist concerning the origin and exact mechanism of release of cfDNA in healthy individuals as well as in tumor patients. It has been reported that in healthy individuals most of the cfDNA originates from (mainly hematopoietic) apoptotic cells 11. Necrosis does not contribute to the cfDNA in healthy individuals 12. However, all living tumor and nontumor cells may also actively release DNA as reported by Stroun et al. in 13. In addition to apoptosis, necrosis of cancer cells, especially those with a high cellular turnover rate, contributes to the frequently observed elevated levels of cfDNA in cancer patients 10,14. It has been suggested that quantification of cfDNA has to be combined with mutation analysis to provide the specificity needed to distinguish between cell-free plasma DNA originating from tumor or nontumor cells 10.

Genetic alterations of oncogenes or tumor-suppressor genes that occur during tumorigenesis provide highly specific markers that allow identification and quantification of circulating tumor DNA (ctDNA) 15. Such tumor-specific mutations have been detected in plasma of patients suffering from various solid cancers or hematopoietic malignancies (for review see 8). Diehl et al. determined the number of adenomatous polyposis coli (*APC*) gene fragments in cfDNA of advanced colorectal cancer patients and found elevated mutant proportions in patients with advanced tumor stages 16 . Later, this group used the same approach to monitor tumor dynamics of colorectal cancer patients undergoing chemotherapy or surgery 17.

Mutations of either *GNAQ* or *GNA11* can be detected in 83% of all (primary or metastatic) uveal melanomas 18. Both oncogenes encode for the alpha subunit of a heterotrimeric GTP-binding protein 19. Activating somatic mutations in both genes can affect codon Q209 (exon 5) or codon R183 (exon 4). *GNAQ* mutations at codon Q209 were found in 45% of primary uveal melanomas, 22% of uveal melanoma metastases, and 55% of blue nevi. Mutations in *GNA11* at codon Q209 were found in 32% of primary uveal melanomas, 57% of the uveal melanoma metastases, and 7% of blue nevi. Mutations at codon R183 of either *GNAQ* or *GNA11* are rare, affecting about 6% of uveal melanomas 18. As a consequence of these mutations, the intrinsic GTPase activity of this alpha subunit is blocked and the protein remains in its active state. The resulting MAP-kinase cascade activation leads to stimulation of cell proliferation, for example, by activation of transcriptional cell cycle genes like *CCDN1* 18,20. Although the MAP-kinase cascade is a mutational target in several tumor entities, activation of this pathway by mutations in either *GNAQ* or *GNA11* is specific for uveal melanomas and other nonepidermic melanocytic lesions like blue nevi 19,20,21. It has been suggested that *GNAQ/GNA11* mutations are present throughout the different stages of the disease and are early events in tumorigenesis 20,22. In this respect, these mutant alleles are suitable markers for detection of ctDNA in plasma of uveal melanoma patients.

Analysis of somatic genetic alterations in cfDNA has been used in many cancers and is a promising tool for noninvasive diagnosis of progressive cancer 15. Several approaches have been used to detect and quantify ctDNA in tumor patients 14,16–23. More recently, ultradeep sequencing technologies have been developed, which enable sequencing of tremendous amounts of DNA fragments in parallel at reasonable cost, thus providing an unbiased view on the ratio of mutant-to-normal reads in amplicons generated on cfDNA from cancer patients 24,25. In particular, the assay can be applied without prior knowledge about the precise nature of the expected genetic alteration.

The goal of our study was to establish an assay for the detection of mutant alleles of *GNAQ* and *GNA11* based on ultradeep amplicon sequencing. We analyzed a consecutive case series of patients with uveal melanoma and extraocular tumor (clinically evident metastases or extraocular growth) to assess if this assay detects ctDNA in these patients.

## Materials and Methods

### Patient samples

This study was approved by the Ethics Committee of the University of Duisburg-Essen (Germany). Informed consent was given by all patients and the Declaration of Helsinki protocols were followed. A consecutive series of 28 patients with a diagnosis of metastatic or extraocular uveal melanoma that had been referred to the University of Duisburg-Essen between November 2010 and September 2011 were asked to participate in this study. Most patients had not received any treatment for metastatic disease at the time of sample collection (see Table 1). Seven patients were under therapy with the multikinase inhibitor sorafenib (varying dosages) and one patient had received intrahepatic chemoembolization 1 month prior to collection of the blood sample. We also included one patient with extraocular growth of the primary tumor who donated blood 3 months prior to clinical diagnosis of metastases. In addition to blood samples, tissue from primary or metastatic tumors was available in nine cases. Plasma samples of seven noncancer individuals were included as negative controls in our study (see Table 2).

**Table 1:** Clinical characteristics of patients and *GNAQ*/*GNA11* mutation status of tumors and cfDNA

ID	Age (years)	Latency PT and M (days)	cfDNA (ng/mL plasma)	Site of metastases at the time of blood sampling	Therapy		Largest diameter (mm)		*GNAQ/GNA11* mutation		
Tumor tissue	Plasma		
PT	M	PT	M	Type	Type	Total reads	Mutant reads (%)
P1	58	773	69	L	E	NT	16.2	82	NA	GNA11 Q209L	2089	3.9
P2	68	803	31	L, LN	B	S	11.2	36	NA	GNA11 Q209L	861	4.2
P3	41	3285	33	L	B	NT	20	111	GNA11 Q209L^1^	GNA11 Q209L	281	4.3
P4	31	869	1550	L, K, LN	B	NT	16.9	54	NA	GNA11 Q209L	3961	38.4
										GNAQ Q209L	4235	2.6
P5	29	4526	82	L, B	Pr	NT	8	101	NA	GNA11 Q209L	1986	21.7
P6	59	448	20	L, B, LN	ER	NT	17.7	30	GNA11 Q209L^1^	GNA11 Q209L	1275	2
P7	49	3150	510	L, B, Mu, LN	B	S	13.7	64	NA	GNAQ Q209L	3588	24.2
P8	75	2774	63	L, B, S	E	S	17.4	77	GNAQ Q209L^1^	GNAQ Q209L	94	6.4
P9	56	346	436	L	B	Ch	12.2	NA	NA	GNAQ Q209P	2951	2.7
P10	49	1249	80	L	B	NT	9.4	48	NA	GNA11 Q209	2523	0
										GNAQ Q209	2701	0
P11	70	2604	18	L	B	NT	13	80	NA	GNA11 Q209L	1212	0.49
										GNAQ Q209	3071	0
P12	65	2564	242	L	B	S	20	35	NA	GNA11 Q209L	3281	0.09
										GNAQ Q209	3395	0
P13	52	457	20	L	E	S	9	39	NA	GNA11 Q209P	1973	0.05
										GNAQ Q209L	3925	0.03
P14	60	2054	132	L, AC	B	S	15.7	15	NA	GNA11 Q209L	2559	0.04
										GNAQ Q209	879	0
P15	52	623	41	L	B	NT	12.9	32	NA	GNA11 Q209	1646	0
										GNAQ Q209P	3150	0.26
P16	56	956	36	L	E	NT	13.8	24	NA	GNA11 Q209	2688	0
										GNAQ Q209P	5313	0.18
P17	59	2841	53	L, Pe	B	NT	11	59	NA	GNA11 Q209L	2601	0.49
										GNAQ Q209	4267	0
P18	70	1222	61	L, SG, ST, Sc, Lu	E	S	15.7	39	NA	GNA11 Q209P	474	0.21
										GNAQ Q209	476	0
P19^3^	78	524	39	–	E	NT	20	NA	GNA11 Q209L^1^,^2^	GNA11 Q209	477	0
P20	75	−13	7	L	NT	NT	20	19	GNA11 Q209^1^	GNA11 Q209L	1442	0.07
P21	55	556	25	L	P	NT	11.7	19	NA	GNA11 Q209L	1549	0.06
GNAQ Q209	3346	0
P22	64	1684	26	L, LN	B	NT	10.8	29.5	NA	GNA11 Q209L	2146	0.09
										GNAQ Q209P	4703	0.02
P23	61	4251	59	L	B	NT	6.4	34	No mutation^2^	GNA11 Q209	Not performed	
										GNAQ Q209		
P24	69	6	14	L, Pa	E	NT	9.8	18.4	GNAQ Q209^1^	GNA11 Q209	Not performed	
										GNAQ Q209		
P25	67	524	98	L, Pa	E	NT	16.4	60	No mutation^1^	GNA11 Q209	Not performed	
										GNAQ Q209		
P26	37	1449	17	L	Pr	NT	17.3	42	NA	GNA11 Q209	Not performed	
										GNAQ Q209		
P27	76	16	37	L, B	E	NT	19	14	GNAQ Q209^1^	GNA11 Q209	Failed repeatedly	
										GNAQ Q209		
P28	76	1411	22	L, Sp, ST, B	B	NT	8.2	35	NA	GNA11 Q209	Not performed	
										GNAQ Q209		

*GNAQ* and *GNA11* ultradeep sequencing in cell-free plasma DNA of metastasized uveal melanoma patients and one patient with extraocular growth of primary tumor.

Age, Age at diagnosis of primary tumor; P, patient; NP, healthy individual; PT, primary tumor; M, metastasis; L, liver; LN, lymph node; K, kidney; B, bone; Mu, muscle; Pa, pancreas; Sp, spleen; AC, adrenal cortex; Pe, peritoneum; SG, suprarenal gland; ST, soft tissue; Sc, subcutis; Lu, lung; E, enucleation; B, brachytherapy; Pr, proton beam irradiation; ER, transretinal endoresection; S, Sorafenib; Ch, chemoembolization; NA, not available; NT, no treatment.

1 Mutation found in primary tumor.

2 Mutation found in metastasis.

3 Patient with extraocular tumor growth, but no metastases at the time of blood sampling, patient developed metastases later on (*GNA11* Q209 positive).

**Table 2:** *GNAQ* and *GNA11* ultradeep sequencing in cell-free plasma DNA of age-matched healthy individuals

ID	Age at blood sampling (years)	cfDNA (ng/mL plasma)	Gene	Total reads	Mutation type	Mutant reads (%)
NP1	33	6	GNA11	3700	Q209P	0
					Q209L	0
				GNAQ	2073	Q209P	0.05
			Q209L	0
NP2	31	4	GNA11	3170	Q209P	0.03
					Q209L	0
				GNAQ	2460	Q209P	0
			Q209L	0
NP3	75	117	GNA11	2301	Q209P	0
					Q209L	0
				GNAQ	1077	Q209P	0
			Q209L	0
NP4	62	8	GNA11	2969	Q209P	0
					Q209L	0.1
				GNAQ	1532	Q209P	0
			Q209L	0
NP5	51	6	GNA11	3841	Q209P	0.05
					Q209L	0.03
				GNAQ	1645	Q209P	0
			Q209L	0
NP6	61	13	GNA11	2764	Q209P	0
					Q209L	0.04
				GNAQ	3875	Q209P	0
			Q209L	0.03
NP7	55	3	GNA11	5421	Q209P	0
					Q209L	0.06
				GNAQ	3743	Q209P	0
			Q209L	0

For legend see Table 1.

### Plasma preparation and cfDNA isolation/quantification

Blood samples were obtained by venipuncture (for clinical characteristics of participating patients see Table 1) using 7.5-mL-sized K-EDTA blood collection tubes (ID 01.1605.001, Sarstedt, Nümbrecht, Germany). The blood was centrifuged at 1500 × g for 10 min within 30 min after sampling. The supernatant (plasma) was collected keeping at least 5-mm distance to the interface and stored at −20°C for later use in DNA preparation. Samples with visual signs of hemolysis (red-colored supernatant) were discarded. Cell-free DNA was isolated from 1–5 mL of plasma using the QIAamp Circulating Nucleic Acid Kit (Qiagen, Hilden, Germany) following the manufacturer's protocol. DNA was eluted in 40 μL AVE Buffer and stored at 5°C. Genomic DNA from primary and metastatic tumor tissue was isolated as described previously 26.

Real-time polymerase chain reaction (PCR) was used to quantify cfDNA 16,23. We used an MGB (minor groove binder) TaqMan assay that targets a genomic 239-bp fragment located in the *AS-SRO* region on chromosome 15 as described elsewhere 27. All samples were analyzed in duplicate.

### PCR reaction and ultradeep sequencing

Amplification of the *GNAQ* Q209 (298 bp), *GNAQ* R183 (212 bp), *GNA11* Q209 (150 bp), and *GNA11* R183 (249 bp) regions was performed using the universal tailed amplicon sequencing strategy as described in the *GS Junior System Guidelines for Amplicon Experimental Design* (Roche, Mannheim, Germany). Briefly, the region of interest was amplified in a first PCR using template-specific primers (for sequences, see 18,19) with a universal sequence at the 5′ end that serves as target for the primers of the second PCR. Different universal tags were used for forward and reverse primers.

In the first PCR, 6 ng of cell-free plasma DNA was used in a final reaction volume of 20 μL containing 0.25 mmol/L of each dNTP, 3.1 mmol/L MgCl_2_ (Applied Biosystems, Darmstadt, Germany), 2.0 μL tenfold Buffer II (Applied Biosystems), 0.5 μmol/L of each primer, and 2U AmpliTaq Gold (Applied Biosystems). After initial denaturation at 95°C for 5 min, the PCR reactions were subjected to 10 cycles of 95°C (20 sec), 63°C (1 min), and 72°C (1 min), followed by 30 cycles of 95°C (20 sec), 56°C (1 min), and 72°C (1 min) and a final extension at 72°C for 7 min. The Univ-A and Univ-B sequences, which are required for the sequencing process on the Roche GS Junior device, were joined to each amplicon in a second round of PCR. Different Univ-A and Univ-B primers, each tagged with a patient-specific multiplex identifier (MID) sequence, were used to provide the ability to sequence multiple samples in a single run. The second PCR was performed in a reaction volume of 50 μL containing 0.15 mmol/L of each dNTP, 3 mmol/L MgCl_2,_ 5 μL tenfold Buffer II, 0.2 μmol/L of each of the primers Univ-A-MID and Univ-B-MID, and 2U AmpliTaq Gold polymerase. After initial denaturation at 95°C for 10 min, PCR was performed for 30 cycles at 95°C (20 sec) and at 72°C (45 sec), followed by elongation at 72°C (7 min). PCR products were separated on a 2% agarose gel and visualized by ethidium bromide staining under UV light. The desired PCR products were extracted from the gel using the QIAamp MinElute gel extraction kit (Qiagen) according to manufacturer's recommendations to get rid of unincorporated nucleotides and primers. Ultradeep amplicon sequencing was performed using a Roche GS Junior sequencing device following the manufacturer's protocol. The GS Amplicon Variant Analyzer software (Roche) was employed to analyze the read data.

Mutation analysis of *GNAQ/GNA11* exons 4 and 5 was performed on DNA from primary or metastatic tumors. Primers and PCR conditions to generate templates for Sanger sequencing were the same as described above for first-round PCR. Sanger sequencing was performed on PCR products purified by gel electrophoresis using one of the first-round PCR primers as sequencing primer. Sequencing reactions, automated electrophoresis, and analysis were performed.

## Results

### cfDNA in plasma

We extracted cfDNA from plasma samples obtained from a series of 28 consecutive patients diagnosed with primary uveal melanoma and either metastatic disease or extraocular extension of the primary tumor (for details see Table 1). Quantification of cfDNA in plasma was performed by real-time PCR targeting the *AS-SRO2* region 27. The *AS-SRO2* amplicon (239 bp) is a suitable reference, as it is similar sized to the *GNAQ* and *GNA11* target regions (150–298 bp). In the metastatic uveal melanoma patient cohort, the results showed a wide range of cfDNA concentrations ranging from 7 to 1550 ng/mL of plasma (median = 40 ng/mL plasma; quartiles: lower quartile = 24 ng/mL plasma; upper quartile = 80 ng/mL plasma). The results in the noncancer cohort showed an overall lower cfDNA concentrations ranging from 4 to 117 ng/mL plasma (Table 2).

### Identification of mutations in exons 4 and 5 of *GNAQ* or *GNA11* in primary or metastatic tumors by Sanger sequencing

Primary tumor or metastatic tissue was available from 9 of 28 patients. We sequenced exons 4 and 5 of *GNAQ* and *GNA11* in DNA from these samples. In seven of nine patients, a somatic mutation was identified (Table 1), each in heterozygous state. The plasma samples from the two patients without mutations in the primary tumor (P23, P25) were excluded from further ultradeep amplicon sequencing.

### Ultradeep sequencing of *GNAQ/GNA11* amplicons from cfDNA

We performed PCR using 6 ng cfDNA, the equivalent of the genome of about 1000 cells. For 3 of the 26 remaining patients (P24, P26, P28), we did not have a sufficient amount of cfDNA needed for deep amplicon sequencing on each of the four amplicons. PCR on cfDNA of one patient (P27) repeatedly failed to produce sufficient PCR product for further analysis. Thus, amplicon sequencing was performed on cfDNA from 22 patients.

Sanger sequencing of tumor DNA had previously shown *GNAQ/GNA11* mutant alleles in 5 of the 22 patients. In three of these five samples, the tumor-specific mutation was detected in cfDNA, albeit with low absolute mutant read numbers (P3, P6, and P8 with 12, 26, and 6 mutant reads, respectively). The tumor-specific mutation was not detected in amplicons of cfDNA of the remaining two patients (P19 and P20), although the number of sequence reads would have permitted detection if it was present at a proportion of over 1%.

Oncogenic *GNAQ/GNA11* mutations were identified in cfDNA of 9 of 22 patients. Mutations were restricted to codon Q209 and affected *GNA11* more often than *GNAQ* (six and four samples, respectively). In most cases, the identified substitution was c.626A>T. A double-nucleotide substitution in *GNA11* (c.626A>T [j] 627G>A) was detected in cfDNA and the primary tumor of one patient (P3). A rare mutation (c.626A>C) that has previously reported in one uveal melanoma only 18 was identified in the cfDNA of patient nine (P9). One patient, P4, showed mutations in both *GNA11* and in *GNAQ* with a proportion of 38.4% and 2.6%, respectively, relative to normal sequence reads.

The proportion of mutant *GNA11/GNAQ* reads obtained from cfDNA varied between patients. In 5 of 9 patients there were <5% mutant reads. Real-time PCR showed no correlation between the proportion of mutant reads and the concentration of cfDNA: the patients with the highest concentrations of cfDNA (P4 and P7 with 1550 and 510 ng/mL, respectively) also showed the highest proportion of mutant reads (38.4% and 24.2%, respectively). However, the patient with third highest cfDNA value (P9, 436 ng/mL) showed the second lowest (2.7%) proportion of mutant reads.

### Clinical findings and mutational status

We compared clinical findings of patients with and without *GNA11* or *GNAQ* mutant alleles in cfDNA as detected by deep sequencing. We found no association to characteristics of the primary tumor, like tumor height or largest basal diameter. However, we observed some relations between the ctDNA mutation status and clinical findings with respect to metastatic disease. First, four of the nine ctDNA-positive patients had metastases in bone, whereas none of the 13 ctDNA-negative patients had metastases at this location (*P* = 0.025, Fisher's exact test). Second, we observed that ctDNA-positive patients were younger at initial diagnosis (mean age 52 years vs. 63 years) and had larger metastases (Fig. 1). Neither the type of treatment of the primary tumor (enucleation, brachytherapy, proton beam irradiation), nor systemic therapy of metastatic disease with multikinase inhibitor sorafenib at the time of blood collection had any discernible effect on the cfDNA mutation status.

**Figure 1:** Diameter of the largest liver metastasis and age at diagnosis in *n* = 8 patients with and *m* = 12 without mutant alleles in ctDNA. Not included are two patients because of missing data and absence of liver metastasis at the time of blood sampling, respectively. Younger patients with larger metastases tended to be ctDNA positive.

## Discussion

We show here that ultradeep amplicon sequencing can be used to detect ctDNA in patients with uveal melanoma and extraocular manifestation. Mutant alleles of the *GNA11* or *GNAQ* genes, which are highly specific for uveal melanoma, were identified in cfDNA of 9 of 22 (41%) patients. Considering that about 80% of primary tumors or uveal melanoma metastases show mutant *GNA11* or *GNAQ* genes 18, it is plausible that only a few of the remaining 13 patients had tumors without one of these mutations, and therefore, were uninformative for our study. In fact, we could not detect any mutant reads in cfDNA (i.e., they were ctDNA negative) in two of five patients with known *GNAQ/GNA11* mutations in the primary tumors. This raises the question why ultradeep sequencing did not detect these mutant alleles in plasma DNA from these patients. One factor known to limit the sensitivity of our assay is the error rate inherent to the next-generation sequencing method that we used 28. Even in healthy individuals, we detected “mutant” reads at a frequency of up to 0.1%. Therefore we took a conservative approach by setting the cut off for detection to 1%, and setting the condition that a mutation has to be detected both in forward and reverse reads. Sequencing errors, however, are very much dependent on sequence context and type of mutation. In fact, the very mutations under study here showed few misreads, and therefore, we could have safely set a site-specific cut off for detection to levels lower than 1% for these mutations. However, applying less stringent cutoff levels to the data obtained from the two ctDNA-negative patients who had *GNA11* mutations confirmed that no mutant reads were evident in their tumor cells (0% and 0.07%). A more general reason that may underlie the failure to detect rare variant DNA is of stochastic nature: presence of only a few mutant DNA molecules in cfDNA increases stochastic bias during early cycles of PCR (PCR drift) 29. This problem was also encountered by Madic et al. 30, who used a very elegant and highly mutation-specific PCR method to detect ctDNA in 20 of 21 patients with metastatic uveal melanoma and known *GNA11* or *GNAQ* mutations 2012. An obvious solution for this problem is to obtain larger sample volumes as this will increase the number of mutant DNA molecules available for study. In addition, the study by Madic et al. suggests that the size spectrum of ctDNA in patients with metastatic uveal melanoma is dominated by smaller sized fragments, analogous to the finding in other tumors 31. Consequently, another possibility to increase the number of amplifiable DNA molecules is to target the PCR primers to smaller regions. This should further increase the sensitivity to detect ctDNA by deep sequencing.

Interestingly, our findings and those of Madic et al. 30 confirm and extend the observation by Raamsdonk et al. (2010) 18 that *GNA11* codon Q209 mutations were more frequent than *GNAQ* codon Q209 mutations in metastatic uveal melanoma than in primary uveal melanoma – of the 12 mutations that we identified in either cfDNA or DNA from metastatic tissue, eight (66%) affected codon Q209 of *GNA11*. The ratios observed by the groups of Madic and Raamsdonk are almost identical with 14/21 (67%) and 13/18 (72%), respectively. In the study by Raamsdonk, metastatic uveal melanoma also showed mutations affecting codon R183 of *GNAQ* and *GNA11* (2/17, 12%). Although none of our patients showed mutations at these positions, it is important to include these positions in the analysis as mutations at these sites are more frequent in metastatic than in primary uveal melanoma.

In one patient (P4), we identified mutations in *GNA11* and *GNAQ* with mutation rates of 38.4% and 2.6%, respectively. Obviously, the cells that contribute to ctDNA in this patient have a heterogeneous *GNA11/GNAQ* mutation status. One possible explanation for this is that the *GNAQ* mutation occurred in a cell that already had a *GNA11* mutation. This would result in a situation where all cells with mutant *GNAQ* are also mutant for *GNA11*, but only some cells with the *GNA11* mutation also show a *GNAQ* mutation, leading to the higher rates of *GNA11* mutation. However, this explanation does not support the observation that *GNA11* mutations tend to be more frequent in advanced tumors 18. Taking this into account calls for another explanation, namely, that the two mutations arose in distinct lineages of tumor cells. Under this assumption, the higher proportion of *GNA11* in ctDNA from this patient indicates a greater contribution of *GNA11* mutant cells to cfDNA in plasma. This would be in line with the greater role of *GNA11* in advanced stages of uveal melanoma.

We found no association between the detection of ctDNA and the size of the primary tumor or treatment modality. This is to be expected, because in all but one patient, the primary tumor had been destroyed months prior to plasma sampling, and thus, it is to be expected that vital tumor cells are present outside of the eye only. We observed that patients with younger age at diagnosis tended to show larger metastases and to be ctDNA positive. Future studies should test if the relation between age at diagnosis and presence of ctDNA is valid. The relation to size was already studied by Madic et al. 30, who found that the amount of ctDNA in plasma correlates well with metastasis volume, which the authors painstakingly determined based on imaging data. We also observed an influence of the site of metastases on ctDNA status. Specifically, all patients with metastases in the bone marrow were ctDNA positive, whereas none of the ctDNA-negative patients had clinically evident metastases at this site. In view of the intimate connection between bone marrow and peripheral blood, such a correlation does not come unexpected, but has not been reported so far to our knowledge.

Detection of ctDNA by ultradeep sequencing has the potential for further development. As the results are counts of specific sequence reads, the relative frequencies of these reads naturally provides quantitative information that can be used to determine ctDNA levels in blood 28. Compared with methods based on allele-specific PCR, ultradeep sequencing covers a broader spectrum of mutations per assay. This is relevant as exemplified by patient P3 in our series, who showed a rare oncogenic *GNA11* mutation (c.626A>T [j] 627G>A) that may not have been detected using other methods. On the downside, the sensitivity of ultradeep sequencing must be improved. However, with recent developments, it has become feasible to distinguish true mutant reads from background noise by paired-end sequencing, and thus, raise sensitivity to one variant in 5000 molecules 28. Certainly, simply taking blood samples and performing ultradeep amplicon sequencing to detect ctDNA would be a very elegant and simple noninvasive method to detect minimal residual tumor disease.

## References

[b1] Singh AD, Bergman L, Seregard S (2005). Uveal melanoma: epidemiologic aspects. Ophthalmol. Clin. North Am.

[b2] Tschentscher F, Prescher G, Horsman DE, White VA, Rieder H, Anastassiou G (2001). Partial deletions of the long and short arm of chromosome 3 point to two tumor suppressor genes in uveal melanoma. Cancer Res.

[b3] Prescher G, Bornfeld N, Hirche H, Horsthemke B, Jockel KH, Becher R (1996). Prognostic implications of monosomy 3 in uveal melanoma. Lancet.

[b4] (2001). Assessment of metastatic disease status at death in 435 patients with large choroidal melanoma in the Collaborative Ocular Melanoma Study (COMS): COMS report no. 15. Arch. Ophthalmol.

[b5] Slattery E, O'Donoghue D (2009). Metastatic melanoma presenting 24 years after surgical resection: a case report and review of the literature. Cases J.

[b6] Damato B (2010). Does ocular treatment of uveal melanoma influence survival?. Br. J. Cancer.

[b7] Kaiserman I, Amer R, Pe'er J (2004). Liver function tests in metastatic uveal melanoma. Am. J. Ophthalmol.

[b8] Anker P, Mulcahy H, Chen XQ, Stroun M (1999). Detection of circulating tumour DNA in the blood (plasma/serum) of cancer patients. Cancer Metastasis Rev.

[b9] Mandel P, Metais P (1948). Les acides nucleiques du plasma sanguin chez l'homme. C. R. Seances Soc. Biol. Fil.

[b10] Jung K, Fleischhacker M, Rabien A (2010). Cell-free DNA in the blood as a solid tumor biomarker – a critical appraisal of the literature. Clin. Chim. Acta.

[b11] Ziegler A, Zangemeister-Wittke U, Stahel RA (2002). Circulating DNA: a new diagnostic gold mine?. Cancer Treat. Rev.

[b12] Suzuki N, Kamataki A, Yamaki J, Homma Y (2008). Characterization of circulating DNA in healthy human plasma. Clin. Chim. Acta.

[b13] Stroun M, Lyautey J, Lederrey C, Mulcahy HE, Anker P (2001). Alu repeat sequences are present in increased proportions compared to a unique gene in plasma/serum DNA: evidence for a preferential release from viable cells?. Ann. NY Acad. Sci.

[b14] Jahr S, Hentze H, Englisch S, Hardt D, Fackelmayer FO, Hesch RD (2001). DNA fragments in the blood plasma of cancer patients: quantitations and evidence for their origin from apoptotic and necrotic cells. Cancer Res.

[b15] Aung KL, Board RE, Ellison G, Donald E, Ward T, Clack G (2010). Current status and future potential of somatic mutation testing from circulating free DNA in patients with solid tumours. Hugo J.

[b16] Diehl F, Li M, Dressman D, He Y, Shen D, Szabo S (2005). Detection and quantification of mutations in the plasma of patients with colorectal tumors. Proc. Natl. Acad. Sci. USA.

[b17] Diehl F, Schmidt K, Choti MA, Romans K, Goodman S, Li M (2008). Circulating mutant DNA to assess tumor dynamics. Nat. Med.

[b18] Van Raamsdonk CD, Griewank KG, Crosby MB, Garrido MC, Vemula S, Wiesner T (2010). Mutations in GNA11 in uveal melanoma. N. Engl. J. Med.

[b19] Van Raamsdonk CD, Bezrookove V, Green G, Bauer J, Gaugler L, O'Brien JM (2009). Frequent somatic mutations of GNAQ in uveal melanoma and blue naevi. Nature.

[b20] Onken MD, Worley LA, Long MD, Duan S, Council ML, Bowcock AM (2008). Oncogenic mutations in GNAQ occur early in uveal melanoma. Invest. Ophthalmol. Vis. Sci.

[b21] Sisley K, Doherty R, Cross NA (2011). What hope for the future? GNAQ and uveal melanoma. Br. J. Ophthalmol.

[b22] Bauer J, Kilic E, Vaarwater J, Bastian BC, Garbe C, de Klein A (2009). Oncogenic GNAQ mutations are not correlated with disease-free survival in uveal melanoma. Br. J. Cancer.

[b23] Gautschi O, Bigosch C, Huegli B, Jermann M, Marx A, Chasse E (2004). Circulating deoxyribonucleic Acid as prognostic marker in non-small-cell lung cancer patients undergoing chemotherapy. J. Clin. Oncol.

[b24] Margulies M, Egholm M, Altman WE, Attiya S, Bader JS, Bemben LA (2005). Genome sequencing in microfabricated high-density picolitre reactors. Nature.

[b25] Bentley DR, Balasubramanian S, Swerdlow HP, Smith GP, Milton J, Brown CG (2008). Accurate whole human genome sequencing using reversible terminator chemistry. Nature.

[b26] Tschentscher F, Prescher G, Zeschnigk M, Horsthemke B, Lohmann DR (2000). Identification of chromosomes 3, 6, and 8 aberrations in uveal melanoma by microsatellite analysis in comparison to comparative genomic hybridization. Cancer Genet. Cytogenet.

[b27] Ronan A, K Buiting, T Dudding (2008). Atypical Angelman syndrome with macrocephaly due to a familial imprinting center deletion. Am. J. Med. Genet.

[b28] Narayan A, Carriero NJ, Gettinger SN, Kluytenaar J, Kozak KR, Yock TI (2012). Ultrasensitive measurement of hotspot mutations in tumor DNA in blood using error-suppressed multiplexed deep sequencing. Cancer Res.

[b29] Wagner A (1994). Surveys of gene families using polymerase chain-reaction – PCR selection and PCR drift. Syst. Biol.

[b30] Madic J, Piperno-Neumann S, Servois V, Rampanou A, Milder M, Trouiller B (2012). Pyrophosphorolysis-activated polymerization detects circulating tumor DNA in metastatic uveal melanoma. Clin. Cancer Res.

[b31] Mouliere F, Robert B, Arnau Peyrotte E, Del Rio M, Ychou M, Molina F (2011). High fragmentation characterizes tumour-derived circulating DNA. PLoS ONE.

